# Analysis of the Current Situation of Teaching and Learning of Ideological and Political Theory Courses by Deep Learning

**DOI:** 10.1155/2022/5396054

**Published:** 2022-08-18

**Authors:** Jin Chao, Yijiang Zhang

**Affiliations:** ^1^Marxist Branch, Shaoxing University Yuanpei College, Shaoxing 312000, Zhejiang, China; ^2^Information and Mechanical and Electrical Engineering Branch, Shaoxing University Yuanpei College, Shaoxing 312000, Zhejiang, China

## Abstract

The objectives are to solve the problems existing in the current ideological and political theory courses, such as the difficulty of classroom teaching quality assessment, the confusion of teachers' classroom process management, and the lack of objective assessment basis in teaching quality monitoring. Based on Artificial Intelligence (AI) technology, a designed evaluation method is proposed for teachers' classroom teaching and solves some problems such as high system cost, low evaluation accuracy, and imperfect evaluation methods. Firstly, the boundary algorithm system is introduced in the research, and the Field Programmable Gate Array (FPGA) by deep learning (DL) is used to accelerate the server hardware network platform and equipped with pan tilt zoom (PTZ) and manage multiple AI + embedded visual boundary algorithm devices. Secondly, the network platform can manage the PTZ and focal length of Internet protocol (IP) cameras, measure, and capture face images, transmit data, and recognize students' face, head, and body postures. Finally, classroom teaching is evaluated, and students' behavioral data and functions are designed, debugged, and tested. The research results demonstrate that the method overcomes the problem of high system cost through edge computing and hardware structure, and DL technology is used to overcome the problem of low accuracy of classroom teaching evaluation. Various indicators such as attendance rate, concentration, activity, and richness of teaching links in classroom teaching are obtained. The method involved can make an objective evaluation of classroom teaching and overcome the problem of incomplete classroom teaching evaluation.

## 1. Introduction

With the development of China's economy and society, language teaching has increasingly attracted people's attention [1]. The quality of language teaching will directly affect the learning effect of students and the quality of personnel training [2]. Classroom teaching evaluation has become an important part of improving the quality of teaching, which is highly valued by educators, and has become a hot topic in teaching research, teaching system reform, and classroom management in colleges and universities [3]. Therefore, it is of great significance to propose an effective and scientific classroom evaluation method [4]. In early high school classroom learning, students' classroom achievements are usually judged by the final exam results. However, this evaluation method cannot fully reflect the students' learning status, nor is it conducive to finding problems and improving education in the process of classroom teaching. It is not conducive to fully mobilizing students' learning enthusiasm [5]. At present, almost all universities adopt a credit system. In some schools, students do not want to learn more professional knowledge but only to obtain enough credits to graduate smoothly. In some classes, there are still phenomena such as playing on mobile phones in class [6].

At present, domestic and international scholars have conducted extensive research on the application of deep learning (DL). Prabakaran and Shyamala proposed a human biometric approach to vocal fingerprints as a unique method for identifying identities. By extracting sound features from digital speech signals and executing them on different platforms, the extracted speech features are tested with different data tools [7]. Zeng et al. studied the optimization of learning algorithms deployed at the edge of the network through edge machine learning, to use massive distributed data and computing resources to train artificial intelligence (AI) models and improve the ability of models to analyze problems [8]. Kumar et al. analyzed that automatic face detection systems play an important role in face recognition, facial expression recognition, head pose estimation, human-computer interaction (HCI), and so on. By studying the differences between various face detection techniques in digital image analysis, the analysis and test situation of different face detection standard databases and their characteristics are finally given [9]. Shen pointed out that there are many problems in modern English education, such as difficulties in classroom teaching quality evaluation, lack of objective evaluation basis for teaching process management, and quality monitoring. The development of AI technology provides new ideas for classroom teaching evaluation, but the existing classroom evaluation schemes based on AI technology have a series of problems, such as high system cost, low evaluation accuracy, and incomplete evaluation. Given the above problems, Shen proposed an English classroom attention evaluation system based on deep learning to evaluate the students' classroom attention, classroom activities, and the richness of teaching links [10].

According to these backgrounds and the requirements in the classroom process management system, a classroom evaluation system based on deep learning (DL) technology is designed and completed. The research will be divided into four parts: the first part is to analyze the research background and relevant research literature; the second part is to combine relevant research theories to design the used methods and systems; the third part is to test the designed method to verify the ability of the method to deal with the problem; and the fourth part is to analyze and summarize the experimental results. Through the innovative method of intelligent scanning, effective classroom full-range monitoring is carried out. DL technology is used to implement semantic-level assessment of classroom teaching, and intelligent assessment and information management of classroom quality are performed.

## 2. Design and Research of Classroom Detection System Based on DL

### 2.1. AI-Based Classroom Recognition Model

The rapid expansion of AI technology has brought new thinking to the classroom teaching evaluation system, and the mature application of DL technology in the field of education has also created opportunities for the realization of a classroom teaching evaluation system that integrates various DL algorithms. Therefore, in the research, it is proposed to design an ideological and political classroom teaching analysis system based on DL technology to analyze the situation of students in the teaching classroom and further supervise the learning situation of students [11]. The system uses DL technology to carry out semantic-level recognition of key signals in classroom teaching and uses the edge computing system as a framework to efficiently perform big data analysis and calculation on the class performance of students. For example, according to factors such as student's attendance, seriousness in class, and interaction with teachers, it is converted into an information-based classroom teaching evaluation index. In the end, a reasonable classroom teaching evaluation and optimization management are carried out.

Tengine is a lightweight, high-efficiency, modular architecture for deepening research on embedded systems [12]. The architecture further optimizes embedded technology equipment based on Advanced RISC Machine (ARM), without relying on third-party databases. It can also be applied across platforms, supports Android, Linux, and so on, and supports the use of Graphics Processing Unit (GPU), Diffusion Limited Aggregation (DLA), and so on, to be used as hardware to increase computing resource heterogeneity [13]. In the in-depth research network supported by Tengine, Multitask Convolutional Neural Network (MTCNN), Solid State Disk (SSD), You Only Look Once-V2 (YOLO-V2), and other networks can provide functions of face recognition [14]. However, because people's real-time demand for face recognition is not very high, the MTCNN algorithm with a slow running speed but higher accuracy is selected to provide face recognition at the edge [15].

The MTCNN mode mainly uses three cascaded network systems, such as Proposal Network (P-Net), Refine Network (R-Net), and Output Network (O-Net) to achieve faster and more effective face data monitoring [16]. This mode also uses key techniques such as image pyramid, border recycling, and off-peak control [17]. P-Net first changes all training samples into the pixel size of 12 × 12 × 3 images and obtains a 1 × 1 × 32 feature map (obtained after convolution) through three convolutional layers. After three different 1 × 1 convolution kernels, three orthogonal protection pixels are obtained, which are 1 × 1 × 2 face probability, 1 × 1 × 4 position of the face candidate frame, and 1 × 1 × 10 five marker determination points of the face [18]. Its network structure is shown in Figure 1.

AI's analytical capabilities have surpassed humans in some aspects. Microsoft's R–Ne is one of the AIs that have reached this milestone. R-Net uses an attention mechanism to highlight certain parts of image features in the context of image analysis. Using Self-Matched Attention helps distinguish the current feature from other features with similar meaning in the rest of the image. R-Net changes each training sample to a pixel size of 24 × 24 × 3. After convolution and pooling, the face probability, the position of the face candidate frame, and the five marker determination points of the face are provided in turn [19]. Its network structure is exhibited in Figure 2.

Output Network (O-Net) changes all training samples to an image scale of 48 × 48 × 3, which is similar to R-Net. However, the provided face probability, the position of the face candidate frame, and the five marker determination points of the face are different [20]. Its network structure is displayed in Figure 3. From P-Net to R-Net to O-Net, as the size of the input image is getting larger and the network structure is getting deeper and deeper, the obtained feature information is more and more expressive [21].

When training the MTCNN network, the following three main tasks must be converged: face probability, the position of the face candidate frame, and the five marker determination points of the face [22]. The following cross-entropy loss function is used for the face, as expressed in

(1) $$\begin{array}{c} L_{i}^{\det}=-\left(y_{i}^{\det}\log\left(p_{i}\right)+\left(1-y_{i}^{\det}\right)\left(1-\log\left(p_{i}\right)\right)\right),y_{i}^{\det}\in \left\{0,1\right\}, \end{array}$$

where *p*_*i*_ represents the sample, *x*_*i*_ is the probability of a face, and *y*_*i*_^det^ expresses the label, which takes a value of 0 or 1.

For the returned results of all candidate boxes, the following sum-of-squares loss function can be used, or the return loss can be estimated using the Euclidean distance, as shown in the following:

(2) $$\begin{array}{c} L_{i}^{\text{box}}=//\hat{y_{i}^{\text{box}}}-y_{i}^{\text{box}}/{/}_{2}^{2},y_{i}^{\text{box}}\in R^{4}, \end{array}$$

where $\hat{y_{i}^{\text{box}}}$ is the coordinates predicted by the network and *y*_*i*_^box^ is the actual real background coordinates; both are quadrupled.

For the marker localization of a face, the following sum-of-squares loss function is used to compute the predicted landmark location and the Euclidean distance of the actual real landmark and minimize this distance [23]. The calculation is shown in the following:

(3) $$\begin{array}{c} L_{i}^{\text{landmark}}=//\hat{y_{i}^{\text{landmark}}}-y_{i}^{\text{landmark}}/{/}_{2}^{2},y_{i}^{\text{landmark}}\in R^{10}, \end{array}$$

where $\hat{y_{i}^{\text{landmark}}}$ is the landmark coordinate predicted by the network and *y*_*i*_^landmark^ is the actual real landmark coordinate. Since there are a total of 5 marker points for the left eye, right eye, nose, left corner of the mouth, and right corner of the mouth, each point has 2 coordinate values, so the *y*_*i*_^landmark^ is a ten-tuple.

Since each network does a different job, different types of training data are required in the process of training. The training equation for multiple input sources is as follows:

(4) $$\begin{array}{c} \min\sum_{i=1}^{N}\sum_{j\in \left\{\det,\text{box},\text{landmark}\right\}}\alpha_{j}\beta_{i}^{j}L_{i}^{j},\beta_{i}^{j}\in \left\{0,1\right\}. \end{array}$$

*N* refers to the number of training samples, *α*_*j*_ represents the importance of the task, *β*_*i*_^*j*^ is the sample label, and *L*_*i*_^*j*^ is the loss function. In the MTCNN, when training P-Net and R-Net, *α*_det_=1, *α*_box_=0.5, and *α*_landmark_=0.5; when training O-Net, *α*_det_=1, *α*_box_=0.5, and *α*_landmark_=1. At last, the network will output three sets of data, which are judgment results of the face/nonface, the coordinates of the upper left and lower right corners of the face frame, and the coordinates of five marker points of the face.

### 2.2. MobileNet-V2

MobileNet-V1, the previous generation network of MobileNet-V2, uses Depthwise Separable Convolution (DSC) technology, which allows the neural network to greatly improve the calculation rate while ensuring accuracy [24]. A new architecture is provided in MobileNet-V2, called Inverted Residuals with Linear Bottlelock. This architecture first increases the dimension of the input feature map by using a 1×1 convolution operation, and then a 3 × 3 convolution method is calculated, and finally the 1 × 1 convolution method is used to reduce the angle. After the convolution is implemented, the Rectified Linear Units (ReLU) activation function will no longer be used, but the linear activation function will be used instead to save more feature signals and improve the expressiveness of the model [25].

To improve the stability of the network system, the linear convolution part in the Inverted Residuals with Linear Bottlelock structure of the network system is adjusted into the Squeeze-and-Excitation (SE) module [26]. An input feature is given, and the number of channels is 1. After a series of transformations, a feature with a channel number of 2 is obtained, and then the feature information is injected into SEBlock, and the new features are obtained after calibration in three steps:

(1) The Squeeze operation uses Global Average Pooling to achieve feature compression along the spatial level, so that each two-dimensional feature path becomes a set of real number spaces, and the input and output levels are consistent with the number of features paths provided. Its expression is shown in the following:
  (5) $$\begin{array}{c} z_{c}=F_{sq}\left(u_{c}\right)=\frac{1}{H\times W}\sum_{i=1}^{H}\sum_{j=1}^{W}u_{c}\left(i,j\right), \end{array}$$
where *u*_*c*_ refers to a two-dimensional matrix and *z*_*c*_ means the output result. H and W represent common parameters.
(2) The Excitation method uses the parameter W to generate weights for each feature path, where the parameter W is used by machine learning to show the relationship between the feature paths. The *z* obtained by multiplying W_1_ by the Squeeze operation is a full connection operation, and through the next ReLU layer, the output dimension does not change [27] and then multiplied by W2, which is also a full connection process. Finally, after passing through the Sigmoid function, weight *s* is obtained. Its expression is shown in the following:
  (6) $$\begin{array}{c} s=F_{ex}\left(z,w\right)=\sigma \left(g,\left(z,w\right)\right)=\sigma \left(W_{2}\delta \left(W_{1}z\right)\right). \end{array}$$
The calculation of parameter W is shown in the following:
  (7) $$\begin{array}{c} W_{1}\in \frac{C}{r}\times C,W_{2}=C\times \frac{C}{r}. \end{array}$$
In equation (7), *r* is a scaling parameter whose purpose is to reduce the number of channels and reduce the computational workload. The dimension of the final output is 1 × 1 × C, where C represents the number of channels. s is used to represent the weight of C feature maps.
(3) After getting *s*, equation (8) is used to operate.
  (8) $$\begin{array}{c} \tilde{x_{c}}=F_{\text{scale}}\left(u_{c},s_{c}\right)=s_{c}\cdot u_{c}, \end{array}$$

where *u*_*c*_ is a two-dimensional matrix and *s*_*c*_ is the weights, equivalent to multiplying each value in the *u*_*c*_ matrix by *s*_*c*_.

The structure of the modified Inverted Residuals with Linear Bottlelock is demonstrated in Figure 4. The network inputs a 128 × 128 image each time and extracts facial feature points and character vectors on the pixel in turn. Finally, a row vector containing 256 floating-point coded values is output, and the row vector is used as the average of the abscissa and ordinate of the facial character vector. The cosine distance between the output characteristic vector value and the characteristic vector position value in the face image is estimated in turn, and the threshold point of the cosine distance is determined. If the cosine distance is lower than the threshold point, the identified face can be determined to be the student himself.

### 2.3. VGG-16

Due to the need for real classroom action recognition of learners in the classroom and there is very little analysis of head-up, expression, and body posture in the recognition process, the recognition results obtained through the Visual Geometry Group-16 (VGG-16) network are better. Therefore, the classroom behavior recognition at the edge is completed through the VGG-16 network system. Open Visual Inference and Neural Network Optimization (OpenVINO) is a development tool suite that helps to improve the development speed of vision applications such as high-performance computer vision and DL. For AI workloads, OpenVINO also provides a Deep Learning Deployment Toolkit (DLDT), which enables the online deployment of all models trained in open source architectures.

DLDT is divided into two parts: Model Optimizer, which is suitable for offline modeling transformation, and Inference Engine which is the AI workload executed by the deployment on the device. In the VGG series network, it is distinguished according to the difference in the size of the convolution kernel and the number of convolutional layers. Among them, the two configurations of VGG-16 and VGG-19 are more commonly used. Tengine supports VGG-16 but not VGG-19, so the system uses the VGG-16 structure. The input data of VGG-16 is an image of 224 × 224 × 3. After passing through the five-layer convolutional network and the pooling network, the output result is a 4096-dimensional feature set, which is then processed by three layers of fully connected layers. Then, the final analysis conclusion is obtained through the Softmax function operation. The Softmax layer dimension can be appropriately adjusted for the number of classifications for various purposes.  Figure 5 indicates the network structure of VGG-16.

## 3. Construction of Classroom Evaluation System

Starting from learner assessment, it has carried out in-depth research on the evaluation methods of teaching engagement, teaching activity, and the richness of classroom teaching links and established an information-based evaluation system for students' learning efficiency and classroom teaching efficiency. The system extracts 10 secondary indicators of classroom evaluation from students' classroom behavior performance, including student attendance rate (A), head posture correct rate (F), head-up rate (H), nonsleep rate (*T*) and teacher explanation (*M*_1_), students taking the initiative to answer questions (*M*_2_), teachers calling and answering questions (*M*_3_), and classroom teaching assignments (*M*_4_). From this, four first-level evaluation indicators are formed, including classroom attendance rate *S*_A_, classroom concentration *S*_F_, classroom activity *S*_V_, and richness of classroom link *S*_M_. Classroom quality evaluation indicators and the weight distribution of each indicator are illustrated in Figure 6.

Classroom evaluation indicators at all levels are calculated on a percentile basis. The weights of the four first-level indicators *S*_A_, *S*_F_, *S*_V_, and *S*_M_ for classroom quality evaluation are represented by W_1_, W_2_, W_3_, and W_4_, respectively. The default values of the system are 70%, 10%, 10%, and 10%, respectively. The specific weight value can be set through the system client interface. Therefore, the score of the system classroom quality evaluation can be calculated by the following:

(9) $$\begin{array}{c} S=S_{A}W_{1}+S_{F}W_{2}+S_{V}W_{3}+S_{M}W_{4},\\ S_{A}=A,\\ S_{F}=f_{1}F_{1}+f_{2}F_{2},\\ S_{V}=v_{1}H+v_{2}R+v_{3}J,\\ S_{M}=X_{1}M_{1}+\max\left\{X_{2}M_{2};X_{3}M_{3}\right\}+X_{4}M_{4}. \end{array}$$

In the calculation process of *S*_M_, only one of *M*_2_ and *M*_3_ is selected, so when *M*_2_ appears, the system does not count the weight of *M*_3_. When *M*_2_ does not exist, the weight of *M*_3_ is only considered.

### 3.1. Camera Distribution in Classrooms and Experimental Design

Existing classroom attendance systems mostly use a single fixed camera to capture images of students in the classroom. Since this solution has only a single camera and a fixed viewing angle, it cannot achieve complete coverage of the classroom area. In addition, there is a solution of using multiple cameras, placing multiple cameras at different positions in the classroom and adjusting different angles to achieve complete coverage of the classroom area. Due to a large number of cameras in this solution, the wiring is relatively more complicated. In response to the above problems, the spherical camera with Pan Tilt Zoom (PTZ) and optical zoom, which is currently equipped in most school classrooms, is used as an image acquisition tool. Through PTZ and focal length control, the entire classroom area can be covered in a fixed position. Since the camera supports optical zoom, it can ensure that the face image is relatively clear while increasing the proportion of the face in the image. Therefore, the face image can be individually captured and adjusted to the minimum resolution that can meet the recognition requirements and then transmitted to the server.

After this processing, more image data can be transmitted with lower bandwidth. Since it is impossible to frame all faces on the screen at one time after zooming, it is necessary to use the PTZ control function of the camera to divide the classroom seats into multiple areas. Control the camera PTZ, so that the camera can collect face images in different areas and can collect all face images in the classroom while ensuring the clarity of the image. The Open Network Video Interface Forum (ONVIF) protocol is used on the Embedded Artificial Intelligence Development Kit-610 (EAIDK-610) development board to control the PTZ and focal length of the camera through the network, so that the camera can capture various areas in the classroom at a fixed position. The image of the students is intelligently scanned, and the efficient monitoring of the whole area of the classroom is realized.

### 3.2. PTZ and Focus Control

According to the scheme of the system design, the school needs to collect images of all student areas in the classroom. The system will use a dome network camera as the video input device. To realize the focal length management of the PTZ for Internet cameras, the ONVIF protocol is introduced. The frame diagram of camera PTZ control is shown in Figure 7.

When managing the PTZ and focal range of the camera, the default gateway for the camera must be first selected to make sure that the camera and the router are in the same gateway. Then, the Internet Protocol (IP) address of the camera is queried, to master the basic information about the camera, including the basic information of various functions supported by the camera. Next, the relevant data information of the PTZ control function is queried from various functional data information, to obtain the technical ability to monitor the dual-camera PTZ and focal length. Finally, the PTZ monitoring parameters are used to monitor the PTZ and focal length.

#### 3.2.1. Face Detection and Face Image Capture

Due to the variable patterns of different faces such as appearance, expression, and skin color, under different circumstances, the presence of accessories such as glasses and beards on the face, as well as the shadow changes generated by the face under different lighting environments, makes the machine unable to detect the position of the face in the image. Therefore, it is necessary to construct a face detection system to monitor the problems of faces in complex environments. Face recognition is a kind of biometric identification technology based on human facial feature information. A series of related technologies collect images or video streams containing human faces through cameras, automatically detect and track human faces in the images, and then perform face recognition on the detected faces. Gesture recognition can come from the movement of various parts of a person's body but generally refers to the movement of the face and hands. Users can use simple gestures to control or interact with devices, allowing computers to understand human behavior.

The system adopts the EAIDK-610 embedded AI application technology research and development (R&D) platform as the image acquisition and neural network computing implementation platform at the edge of the system. The date of the operating system on the EAIDK-610 development board is adjusted to be the same as the school date. Adding a timing start command before the corresponding program of the attendance function allows the system to automatically execute the attendance program from the beginning of each class. While measuring the faces of the students, the system will also record the coordinates of the seats of the students in the classroom, bind the coordinate values to the name of the captured face image, and then load another statistical data file. After the face recognition is successful, the student information will be matched with the coordinate value, which is convenient for classroom management of each class in the future. The frame diagram of the face detection and face image capture functions is displayed in Figure 8.

#### 3.2.2. Classroom Behavior Recognition

In the class stage, after the first attendance check is completed, restore the camera PTZ, add the head-up recognition mode, head posture recognition mode, expression recognition mode, and body posture recognition module on the EAIDK-610 development board, and start to recognize the real classroom behavior of each student in the classroom. The framework of classroom behavior recognition is shown in Figure 9.

In Figure 9, for head-up recognition, there are two classification results of “head-up” and “non-head-up.” For head posture recognition, there are two classification results of “looking at the podium” and “not looking at the podium.” For human posture recognition, there are five classification results of “sitting down,” “standing,” “raised hands,” “writing,” and “sleeping.”

## 4. Results and Discussion

Based on the analysis of functional requirements, the designed course evaluation system based on DL will have the functions of course attendance, teaching behavior recognition, classroom teaching quality evaluation, and learners' classroom behavior statistics. The test is mainly carried out in the laboratory, and a total of ten people participate in the test. In addition to the two attendance tests, a total of 80 classroom behavior recognition test time points are set, and the diagram of attendance in the database is shown in Figure 10.

After the camera collects pictures of a certain range, it will frame the faces of all students with a yellow frame. When the camera stays in this area for three to five seconds, it will capture all the students' face pictures in the yellow frame, adjust the length to 128 × 128, and store them in the storage port of EAIDK-610 in sequence. After testing, the designed system has realized the function of classroom attendance.

### 4.1. Classroom Evaluation and Statistics of Students' Classroom Behavior

The diagram of classroom evaluation in the database is shown in Figure 11.

Figure 11 shows the results of head posture recognition performed by the camera on the student in the seat. Since the system has set a total of 80 detection time points for head posture recognition, there are a total of 80-time points data on the number of students looking at the podium in the results of head-up recognition after the teaching is completed. At the same time as completing the recognition of human posture, since the system records the status of students' raised hands and sleep status, there will also be data on the number of students who raised their hands and the number of sleepers at the corresponding time point after the teaching is completed. Grades are uploaded to the appropriate place in the classroom grading table in the database.

Meanwhile, the statistical analysis results of all students' class situations are also uploaded to the corresponding place in the statistical analysis table of students' class situations in the database system. The statistical graph of the student's classroom behavior in the database is shown in Figure 12.

In Figure 12, the height of the histogram reflects the time proportion of various classroom behaviors during the students' class. Most students can seriously participate in the class. After testing, the designed system has realized the function of classroom evaluation. According to the generated evaluation chart of students' classroom behavior, it is very clear to understand the performance of each student in the whole class process, which is very helpful for the reward and punishment of students' performance in the later stage.

### 4.2. Design of Performance Test of the System

To verify the effectiveness of the design method to deal with the problem, the designed algorithm is used to test face detection, face recognition, gesture recognition, and other situations. The test results using the VGG-16 network during the experiment are illustrated in Figure 13.

In Figure 13, the face detection rate has reached 90%, the face recognition rate has reached 94%, and the posture recognition has reached 80%. The face detection test can be realized through the MTCNN. Through the network system with MobileNet-V2 as the backbone, face recognition and detection are realized. The research results manifest that according to the characteristics of the system design, the various factors affecting the system characteristics are divided into face feature detection efficiency, face recognition efficiency, head posture recognition rate, head-up recognition rate, expression recognition rate, body posture recognition rate, system stability, and so on. It can improve the ability to design algorithms to analyze problems.

## 5. Conclusion

Based on the system functional requirements and design requirements, the overall research process of the DL-based classroom evaluation system is introduced in detail from the aspects of system scheme design, related calculation, and detailed design. The designed classroom teaching evaluation system has been tested for function and characteristics. Firstly, starting from the background of DL and classroom evaluation system, the research objectives are given for the problem, and then the overall scheme of the system is designed. Secondly, based on the research background and actual usage scenarios, the decomposition of the system functional requirements is carried out, and the system design requirements are further clarified. On this basis, the overall scheme design of the system as well as the construction scheme design of the hardware platform and the software system is given. Then, the network platform can manage the PTZ and focal length of IP cameras, detect and recognize faces, transmit data, recognize faces, and recognize students' postures and other behaviors. Finally, through the experiment, the design, debugging, and testing of related functions such as teaching evaluation and student behavior statistics are carried out, and the detailed design of the system is completed.

The experimental results manifest that the system achieves the expected effect, and all the main performance parameters meet the design conditions. However, due to the limitations of the times and space conditions, there are still many aspects to be added and improved. The optimization of the CNN and the realization of the specific functions of the classroom evaluation part of the education system still need to be further improved. Moreover, the data set samples used in the research also need to be improved, and a more comprehensive sample data set needs to be established to improve the effectiveness of model training. In the follow-up research, aiming at these problems, the experimental process and the designed model will be further optimized, which will play a guiding role in the future research direction.

## Figures and Tables

**Figure 1:** The network structure of P-Net.

**Figure 2:** The network structure of R-Net.

**Figure 3:** The network structure of O-Net.

**Figure 4:** The structure of the modified Inverted Residuals with Linear Bottlelock.

**Figure 5:** The network structure of VGG-16.

**Figure 6:** Classroom quality evaluation system.

**Figure 7:** The frame diagram of camera PTZ control.

**Figure 8:** The frame diagram of the face detection and face image capture functions.

**Figure 9:** The framework of classroom behavior recognition.

**Figure 10:** The diagram of attendance in the database.

**Figure 11:** The diagram of classroom evaluation in the database.

**Figure 12:** The statistical graph of the student's classroom behavior in the database.

**Figure 13:** The results of each test.

## Data Availability

The data used to support the findings of this study are included within the article and more detailed data used to support the findings of this study are available from the corresponding author upon request.
